# A Deep Learning-Based Piano Music Notation Recognition Method

This article has been retracted.

**DOI:** 10.1155/2022/2278683

**Published:** 2022-06-02

**Authors:** Chan Li

**Affiliations:** School of Preschool Education, Guangdong Nanhua Vocational College of Industry and Commerce, Guangzhou 510510, China

## Abstract

In the era of rapid development of computer technology, piano music notation and electronic synthesis system can be established using computer technology, and the basic laws of music score can be analyzed from the perspective of image processing, which is of a great significance in promoting piano improvement and research and development, etc. In this paper, the Beaulieu analysis method is used to analyze the piano music notation and electronic synthesis system module. For piano sheet music, sheet music recognition is the main problem in the whole system. Through the digital recognition method, the piano sheet music feature matrix is extracted to get the piano sheet music multiplication frequency points and the envelope function needs to be extracted for better electronic synthesis of piano sheet music. The envelope function can represent the relationship between piano sound intensity and time change and finally achieve the recognition of the piano score. We extract the music information from the digital score, thus converting the music information into MIDI files, reconstructing the score, and providing an audio carrier for the score transmission. The experimental results show that the system has a correct rate of 94.4% in extracting music information from piano scores, which can meet the needs of practical applications and provide a new way for music digital libraries, music education, and music theory analysis.

## 1. Introduction

In the era of rapid development of computer technology, music and electronic synthesis are widely concerned by musicians, and the use of computer technology allows for the creation of piano music notation and electronic synthesis systems, which are important to promote the improvement and development of the piano, among other things [1]. With the advancement of electronic synthesis technology, computers are producing electronic synthesis scores, especially for the piano, which are very beautiful, and with electronic synthesis, more new scores will appear that perfectly demonstrate the uniqueness of the piano and its application to computer music composition. Computer technology for piano notation and electronic synthesis plays an important role in electronic music; however, computer technology is an important method to achieve piano music notation and electronic synthesis [2, 3].

Piano is a keyboard instrument used in various countries. The sound range of the piano is very wide, and the recognition of piano music symbols is very important [4–6]. The design of the piano music score and the electronic synthesis system based on the improved linear modulation method is proposed. This method separates harmonic signals according to the edge tone of piano music, transmits the music score, analyzes the continuity of the piano music score signal, and completes the design of the piano music score and the electronic synthesis system, but the performance of this method is poor [7, 8]. The method proposes the design of the piano score setting and the electronic synthesis system based on the audio tampering method, extracts and measures the piano score, enhances the characteristic parameters of the piano score, classifies it, judges whether the score has been tampered, compares the authenticity of the score, and finds that the accuracy of this method for the piano score is low [9–12].

The rapid development and popularity of digital technology and network technology have provided material conditions for the conversion of paper sheet music into music sound dissemination; however, the key problem to be solved is how to digitize the sheet music, convert the paper sheet music into digital sheet music, and automatically generate the corresponding digital audio to realize the dissemination of music on the Internet. Currently, there are two main methods to realize digital scores: one is to manually input the scores into computers by music professionals through music software (e.g., Cakewalk, etc.), which relies on professionals and has low work efficiency; the other is to use OMR (optical music recognition) technology for an automatic input [13, 14]. OMR integrates image processing, pattern recognition, artificial intelligence, MIDI, and other related technologies and can convert scores within seconds, which greatly improves the work efficiency and is widely used in digital media music libraries, large digital music libraries, reading and playing of robotic scores, computer music teaching, music teaching, and digitization of traditional Chinese scores [15–18].

## 2. Knowledge in the Field of Music Notation

Notation is a method of recording musical scores. In the course of music development, various notation methods have been created due to the different contents and needs of the music, such as the guqin score for the guqin, the gong score for the gongs and drums, and the five-line score, the short score, and the kongjue score used in our folklore [19]. Notation is very important for creation and performance. Notation must be able to record all aspects of musical activities, including the height, strength, length, musical notation, and expression marks. Notes are symbols that record the progression of notes of different durations [20]. A rest is a symbol that records the interruption of a note of different lengths. In western notation, the common notes and rests are shown in Figure 1.

## 3. Extraction of Musical Information from Digital Sheet Music Based on Mathematical Morphology

The workflow of digitizing paper sheet music and extracting music information based on the OMR system is shown in Figure 2.

The following is an example of a polyphonic piano score using mathematical morphology to process the digital image of the piano score and extract the musical information from the score. It is unrealistic to extract all the musical information of the score, and the purpose is only to get the sound corresponding to the score, so it is not necessary to identify the large number of performance cues in the score (the sound is originally the result of the performance). However, the basic note pitch, time value, and polyphony must be identified. By combining their information, the sound file (MIDI file) corresponding to this score is created, and the score can be reconstructed using the MI-DI file, as shown in Figure 3.

In the image preprocessing stage, because the background of the pentatonic image is single and the color used for recording music information is single, the binarization image processing technique can be used to transform the paper pentatonic into a binary image, and at the same time, the pepper-like restless sound is removed by using the mathematical morphology of first erosion and then expansion operation [21, 22].

Let the image to be processed be *A*, its height be *H*, and its width be *W*.

In the music information recognition stage, the Y-projection technique (horizontal statistics) is used to obtain the information of the music score lines. The number of black pixels in each line is counted as a statistical unit, and the array *s*[*n*], 1 ≤ *n* ≤ *W* is obtained. If the value of each element in *s*[*n*] is considered as a grayscale value, the grayscale histogram, called the numerical histogram, can be counted. Obviously, there are two peaks in the numerical histogram, from which we can get the threshold value that divides the two peaks, denoted as *f*, find the elements in the array *s*[*n*] that are greater than *f*, denoted as a total of *m*, get the sequence of subscripts of these elements, denoted as *R*_*i*_, and satisfy 1 < *R*_*i*_ < *W*1 ≤ *i* ≤ *m*, *S*[*R*_*i*_] > *f*.

Let the width of the spectral line be *k*; obviously, there is *k* ≥ 1, and there is the property.

If *k*  = 1, then *R*_*i*+1_ − *R*_*i*_ ≤ 1,1 ≤ *i* > *m*; if *k* > 1, then, there exists *i*, which satisfies *R*_*i*+1_ − *R*_*i*_=1,1 ≤ *i* < *m*, *t*, *D*.

Note that there are *t* different *i* satisfying conditions *k* > 1 and *R*_*i*+1_ − *R*_*i*_=1.

The distance between spectral lines is defined as *d*:

(1) $$\begin{array}{c} d=\frac{\left.\sum_{i=1}^{m-1}\left(R_{i+1}-R_{i}\right)\right.-t}{m-t}. \end{array}$$

In this paper, a fragment of Beethoven's “Turkish March” (digital image A) was selected for processing, and the results are shown in Figure 3, where the digital image of the score is shown on the left, the corresponding part on the right is the result of *Y*-projection, and the numerical histogram is shown on the upper right.

The score and key number can be identified by using the hit and miss operation based on the position of the score line and the distance *d* from the score line.

The note can be identified using the erosion operation. Let *B*1 be a structural element consisting of black pixels of (*d* − *k*)*∗*(*d* − *k*), and using the erosion operation, the note head can be identified and the position information of the note head can be obtained.  Figure 4 shows the result of the erosion of Tchaikovsky's “Four Little Swans,” where the pitch of the note is determined based on the position of the score and the note head. Also, by setting *B*2 as a structural element consisting of 1*∗*[4*∗d*+3*∗k*] black pixels, the stem and bar line of the notes can be obtained by the corrosion operation.  Figure 5 shows the corrosion result of Beethoven's “For Alice” [23, 24].

The two operations *A*Θ*B*1, *A*Θ*B*2 can be performed in parallel, and the relationship between the note head position and the note stem position is used to design the structural elements *E* and *F*. Using these two structural elements, the temporal information of the notes can be obtained by hitting the hit-miss transformation of the score image.

After getting the complete note information, all the notes are divided into bars by bars using bar lines, and each note belongs to one bar only, and the time values in all bars are calculated to determine whether they are equal or not.

Finally, the extracted music information is combined and converted into MIDI files according to the data structure of the MIDI 1.0 protocol.

## 4. DC-CNN-Based Music Notation Recognition Model

The reduction model proposed in this paper adopts a multilayer convolutional stacking and gate activation function model without a pooling layer similar to PixelCNN. The model is based on an extended causal convolutional neural network (DC-CNN), and the reduction features are introduced by controlling the gate activation unit of each neuron in the neural network to achieve the reduction of electronic artifacts. The DC-CNN adopted in the model exists in causal convolution and expanded convolution, and the DC-CNN has achieved good results in the speech synthesis model WaveNet [25, 26].

### 4.1. Expanded Causal Convolutional Neural Network (DC-CNN)

Generally, each neuron of a convolutional neural network (CNN) consists of a feature extraction layer responsible for extracting the local features of the previous neuron and a feature mapping layer consisting of multiple feature-mapping planes together required during the computation of that neuron.

As shown in Figure 6, the expanded convolution is combined with causal convolution to form an expanded causal convolutional neural network (DC-CNN). This network can control the speech data to be transmitted backward in an orderly manner in time order but also can expand the perceptual field without increasing the number of layers of the neural network and the size of the convolutional kernel, which makes it have excellent performance in processing speech signal data.

### 4.2. Structure of the DC-CNN-Based Music Notation Recognition Model

The speech signal *x*_*T*_ is predicted to be reduced by the input speech signal before time *T* with the reduction factor *h*. The multidimensional joint variable distribution of speech signal sequences *X*=(*x*_1_, *x*_2_, ..., *x*_*T*_) over a period of time can be expressed as

(2) $$\begin{array}{c} P\left(X\right)=\prod_{t=1}^{T}P\left(x_{t}|x_{1},x_{2},...,x_{t-1},h\right). \end{array}$$

As shown in Figure 7, in order to make the music notation recognition sequence generated with the aforementioned conditional probability, the neural network body of the DC-CNN-based music notation recognition model is modeled with a multilayer stack of expanded causal convolutional blocks and a nonlinear mapping is achieved by introducing a gate activation function.

## 5. Experimental Analysis

A server with a Xeon(R) E5-2620 processor and an NVIDIA Quadro M4000 high-performance computing unit was used to train a reduced model with a 20-layer convolutional neural network. The 20-layer convolutional neural network is divided into 2 convolutional blocks, and the expansion coefficients in each block are (20, 21, 22,…, 29) in order. The size of the perceptual field in the reduced model is 128 ms, the number of connected channels in the leap layer is 256, and the initial learning rate is set to 10-3. 869 audio segments are selected for the training set, and the test set consists of 2 piano pieces and 503 English speech segments, all of which are sampled at 16 kHz and quantized at 16 bits [27–30].

The average training time per iteration was 5.0316 s for the piano piece and 3.7273 s for the English speech, and the average training time per 1 s speech was about 36.15 s.

### 5.1. Acoustic Features for Music Notation Recognition

The broadband speech spectrograms of the reduced piano piece and English speech are extracted, and the speech spectral envelope structure is observed, and the vocal pattern features are analyzed. As shown in Figure 8, the restored piano piece is weak in noise, with good audio continuity and a high restoration rate in the low-frequency part.

By comparing the broadband spectrograms of piano pieces with those of English speech, we can see that the broadband spectrograms of the model-reduced speech are clear, with obvious waveforms and high reduction rates.

### 5.2. LPC Data Analysis for Music Notation Recognition

Linear predictive coding (LPC) was first applied to speech analysis and synthesis by Itakura et al. in 1967 and has been widely used in speech signal processing technology since then.

As shown in Figures 9 and 10, LPC data were analyzed separately for the reduced piano music and English speech and the resonance peaks of the music notation recognition and the original speech were consistent with each other; the positions of the resonance peaks generally matched, with only deviations in the intensity of the sound. In Figures 9 and 10, the black solid line and gray solid line indicate the LPC data of music notation recognition and original speech, respectively.

The deviation between the arithmetic mean of music notation recognition and the arithmetic mean of the original speech was calculated for these main parameters. From Table 1, it can be seen that the center frequencies of the musical notation recognition of piano pieces and English speech are very close to their corresponding original speech, and the absolute average deviations of the two are 3.79% and 0.97%, respectively; the intensity of the sound is the second, and the absolute deviations of each artifact are within 13%. Only the bandwidth has a certain degree of deviation.

The analysis results prove that the proposed reduction model can achieve high-quality resonance peak waveform recovery; the overall reduction fit rates of the resonance peak parameters of piano music and English speech reach 79.03% and 79.06%, respectively, which are 44.03% and 44.06% higher than the 35% similarity ratio between the electronic artifact speech and the original speech, respectively.

### 5.3. Human Audiometric Identification of Sameness for Music Notation Recognition

In addition to the electroacoustic instrumentation, 15 volunteers were invited to conduct human ear audiometry to identify the identity of the electronic artifacts and music notation recognition of piano pieces and English speech, respectively, with their corresponding original speech. In the statistical results listed in Table 2, the percentage of identity between the musical notation recognition and the corresponding original speech for piano and English speech increased significantly compared with the percentage of identity between the electronic artifacts and their corresponding original speech, with a maximum increase of 46.67% and a minimum increase of 26.66%, indicating that the reduction model can effectively reduce the electronic artifacts in the speech and make the musical notation recognition. This indicates that the reduction model can effectively reduce the electronic artifacts in the speech and make the music notation recognition closer to the original speech in terms of human ear primary observation.

Due to the influence of noise, the human auditory recognition results of music notation recognition differed from the vocal pattern characteristics and LPC data analysis, so the percentage of volunteers judged the same source as the original speech during human auditory recognition for the noisy music notation recognition was low. In addition, the quality of the music notation recognition was affected by the *μ* − law compression and amplification conversion of the original speech and the auditory effect was not good, which made some of the audio less effective in the human auditory recognition experiment.

## 6. Conclusion

With the advancement of electronic synthesis technology, computer technology for piano notation and electronic synthesis plays an important role in electronic music but also in various musical themes. In this paper, we analyze and study the piano score and electronic synthesis system module using the Beaulieu analysis method. We extract music information from digital scores, thus converting music information to MIDI files, reconstructing the score, and providing an audio carrier for score transmission. The experimental results show that the system has a correct rate of 94.4% in extracting music information from piano sheet music, which can meet the needs of practical applications and provide a new way for music digital library, music education, and music theory analysis.

## Figures and Tables

**Figure 1:** Common notes and rests.

**Figure 2:** Music information extraction process based on the OMR system.

**Figure 3:** Example of *Y*-projection results and their numerical histograms.

**Figure 4:** The score (a) and the result of the corrosion operation of *A*Θ*B*1(b).

**Figure 5:** The score (a) and the result of the corrosion operation of *A*Θ*B*2 (b).

**Figure 6:** Schematic diagram of the expanded causal convolutional neural network.

**Figure 7:** Structure of the DC-CNN-based music notation recognition model.

**Figure 8:** Broadband speech spectrogram of music notation recognition and original speech (partial).

**Figure 9:** Graph of LPC data analysis of music notation recognition of piano pieces with original speech (partial).

**Figure 10:** Graph of music notation recognition of English speech with LPC data analysis of original speech (partial).

**Table 1:** Deviation of main parameters of music notation recognition and the original speech (unit: %).

Audio	Parameters	Pitch	Rate	Tempo
Piano music	Center frequency	6.29	4.50	0.59
	Bandwidth	26.01	66.69	63.95
	Intensity	−9.99	0.65	−10.12

Overall absolute deviation = 20.97 overall reduction fitting rate = 79.03				
English pronunciation	Center frequency	0.50	−2.11	−0.36
	Bandwidth	49.33	72.01	29.55
	Intensity	−11.22	−10.98	12.88
Overall absolute deviation = 20.97 overall reduction fitting rate = 79.03				

Note: overall restoration fit rate = 100% − overall absolute deviation.

**Table 2:** Speech homogeneity human ear audiometric recognition(unit: %).

Audio	Identity identification	Pitch	Rate	Tempo
Piano music	Electronic camouflage voice	33.22	20.00	45.69
	Restore voice	74.44	60.00	80.11
	Improve proportion	41.01	39.09	33.29

English pronunciation	Electronic camouflage voice	26.68	20.00	26.79
	Restore voice	54.44	67.01	74.44
	Improve proportion	26.77	46.47	47.67

## Data Availability

The experimental data used to support the findings of this study are available from the corresponding author upon request.
